# Research on Resource Allocation and Optimization of Community Intelligent Sports Service for the Elderly Based on Group Intelligence

**DOI:** 10.1155/2021/1185533

**Published:** 2021-12-21

**Authors:** Qiaofeng Liu, Jinglun Huang, Bin Zhang, Jihong Zhao, Chengyun Zhang, Xiang Gao

**Affiliations:** ^1^Guangzhou Sport University, Guangzhou 510500, China; ^2^Bangkok Thonburi University, Bangkok 0066, Thailand; ^3^Guangdong Ecological Vocational College, Guangzhou 510500, China; ^4^School of Physical Education, Chaohu College, Hefei Anhui238000, China; ^5^Guangdong Engineering Vocational and Technical College, Guangzhou 510500, China; ^6^Guangdong Judicial Police Vocational College, Guangzhou 510500, China

## Abstract

*Objective.* The mainstream development trend in the era of intelligent sports. At present, with the rapid development of science and technology, it is absolutely wise to combine group intelligence with community intelligent sports services for the elderly. Group intelligence has opened a new era of intelligent sports service. Group intelligence has become an important factor in the development and growth of community intelligent sports service for the elderly and has become a hot topic at present. However, intelligence has encountered difficulties on the road of development. At present, the aging of the population is getting worse and worse, and the elderly have higher and higher requirements for fitness and leisure services, which leads to the need for sports services to be continuously strengthened. The distribution of resources is uneven, the data is not clear enough, and the swarm intelligence algorithm is not perfect. With the adaptation of the elderly to intelligence, more intelligent, concise, and personalized services need to be developed. The most important method is to optimize the swarm intelligence algorithm continuously. In this paper, PSO algorithm is optimized and HCSSPSO algorithm is proposed. HCSSPSO algorithm is a combination of PSO algorithm and clonal selection strategy, and test simulation experiments, PSO algorithm, CLPSO algorithm, and HCSSPSO algorithm for comparison. From the experimental results, HCSSPSO algorithm has better convergence speed and stability, whether it is data or comparison graph. The data optimized by HCSSPSO algorithm is higher than the original data and the other two algorithms in terms of satisfaction and resource allocation.

## 1. Introduction

At present, people pay attention to the development of science and technology, and at the same time, they also pay attention to the development of sports services for the elderly. Since 2013, group intelligence has opened a new door to the development of sports. Up to now, group intelligence has created a lot of value for sports services for the elderly. With the addition of swarm intelligence, the research on sports service for the elderly has been deepened by experts, and the entry of computer intelligent algorithms and analysis methods has completely changed the original traditional sports service mode for the elderly. With the arrival of the new model, the data sources are more extensive, the data is more accurate in this province, and a qualitative leap has been made fundamentally. In this way, the service structure is no longer single but diversified. The elderly are no longer affected by time, weather, and geographical location, which enables the elderly to participate in community sports and enjoy the services brought by science and technology at will, greatly improving the sports level and enthusiasm of the elderly, and enabling smart sports services to continuously absorb suggestions and continuous optimization and improvement.

Literature biology is the origin of swarm intelligence [1]. After continuous development, a group of uncomplicated agents or groups have become swarm intelligence systems. The emergence of “intelligent” global behavior is not known to individuals because its agent interaction follows the principle of locality and randomness. This means that biologists and computer scientists are obsessed with the complex and self-coordinating groups [2]. Out of individual behavior and interaction, flocks of birds, fish, and social insects show problem-solving skills. In the field of swarm intelligence, the development of new algorithms is closely related to biological behavior. Since 1990s, optimization problems in various fields have been solved by animal-based swarm optimization methods [3]. However, the optimization and deepening of swarm intelligence algorithm require continuous research on biological intelligence behavior. Up to now, swarm intelligence can be summarized into three parts. From the biological basis, scientists have obtained the operating principles in biological systems [4]. From the artificial literature, two basic analysis methods and group model techniques are provided and summarized. From the point of view of swarm engineering, Kazadi is the application foundation, and at the same time, swarm intelligence is dominant in a series of applications such as robot system. Similarly, because of the extensive development of swarm intelligence, it is also excellent in solving some theoretical problems [5]. There are many swarm intelligence algorithms, and particle swarm optimization is one of them. Particle swarm optimizer was invented by this algorithm. The random velocity of particles will deeply affect the arrangement of particles according to their unique values, and the addition of mutation factor can keep the balance of pBeat locality values. Therefore, the optimized particle swarm optimizer has great advantages in solving constraint satisfaction problems like *n* queen problem. It is not only a theoretical problem, but also an excellent solution to practical problems [6]. According to the ant colony optimization technology in swarm intelligence, a network framework suitable for the performance factors of small satellites can be constructed. This network framework is different from the traditional network communication architecture and can realize various functions among small satellites more. From the results, it can be seen that the factors of the proposed frame motion change are very consistent. At the same time, it shows that the network topology is not fixed and unadaptable, and it can be transformed to be changeable and adaptable under certain conditions. The necessity of transforming the knowledge of swarm intelligence algorithm effectively needs to be confirmed by considering the brain [7]. In the aspect of development science, the construction of framework is the basis of developing swarm intelligence algorithm, so as to realize the development and evolution of algorithm. However, there are serious problems in the current society, and the aging problem continues to worsen [8]. In order to avoid the weaknesses brought by the traditional old-age care model, a new smart community old-age care model has emerged. This smart community model is based on BCG and provides solutions for changing the original rigid, single, and crude social old-age care services. With the aggravation of population aging, people have higher requirements on the issue of providing for the aged [9]. With the rapid development of science and technology in today's society, people are willing to use science and technology to solve problems and improve schemes. The combination of old-age care and science and technology has become a matter of course and has been widely concerned. However, at present, the market development only considers the ability and needs of the elderly unilaterally, and interactive design is the most prominent aspect. In order to get a suitable interactive design of intelligent aged care services, we must fully consider the needs of the elderly in all aspects and correct the existing intelligent service problems. According to the survey [10], the service level of basic community sports for the elderly is still not high, and there is a high and low gap between urban and rural areas. As the main body of community sports, the satisfaction of the elderly is the future development of community sports [11]. From the aspect of facilities, satisfaction is deeply affected by equipment. From the aspect of sports management, men and women, as well as the elderly in different regions, are obviously satisfied with the first two aspects. From the perspective of education, the fluctuation of satisfaction is gentle under the influence of education. From the aspect of natural environment, the satisfaction degree in each dimension of environment is related to different ages. Community elderly service system is in a series of problems, and the solution can be found in the reform of community sports service management system and professional guidance [12], and laws, venues, facilities, resources, and other aspects should be strengthened. Because the elderly are old, their legs and feet are inconvenient, and their sports level is generally not high. Similarly, their satisfaction with community sports scores is the same [13]. The higher the satisfaction degree of the elderly for community sports including environment and equipment, the higher the willingness of the elderly to participate in community sports. The more the community sports activities and professional guidance, the more the elderly participate in community sports. Therefore, only by paying more attention to and improving the above factors can we strengthen the sports behavior of the elderly. From the perspective of the elderly themselves [14], after receiving physical education, the way the elderly use portable smart devices and the ease or difficulty of perceiving this behavior are important factors that positively affect their behavior intentions. The social pressure that the elderly feel about whether to use this kind of equipment is the main reason that negatively affects their behavioral intention, and the way that the elderly use this kind of equipment balances the social pressure and behavioral intention that the elderly feel. All in all [15], the traditional way of fitness will be broken by the Internet of Things, and this new technology will change the world outlook after the Internet. Smart sports are studied based on the Internet, and a series of effective measures to improve the overall physical fitness of the elderly are discussed. At the same time, the development of intelligent sports for the elderly in the community will be deeply analyzed and studied. As a product of smart sports, the information collected by smart devices will be uploaded to the database, analyzed and processed centrally, and managed properly. In this paper, PSO algorithm is optimized and HCSSPSO algorithm is proposed. HCSSPSO algorithm is a combination of PSO algorithm and clonal selection strategy. The PSO algorithm, CLPSO algorithm, and HCSSPSO algorithm are compared by experiments. HCSSPSO algorithm has good convergence speed and stability in both data and comparison graph. The data optimized by HCSSPSO algorithm is higher than the original data and the other two algorithms in terms of satisfaction and resource allocation.

## 2. Analysis of Swarm Intelligence Algorithm

### 2.1. Basic Concepts

In order to use space, some different kinds of animals will live together, and they are often more complex than other animals. At the same time, this lifestyle means high efficiency and strong creativity. Scientists have taken a fancy to this property, thus developing swarm intelligence [16]. It is precisely because of this property that the control of swarm intelligence is decentralized. Individual behavior in a group will affect other individuals, resulting in a new behavior pattern. There are five basic principles of swarm intelligence. First, all time and space can be calculated without complexity and follow the proximity principle. Secondly, the change of quality factor is closely related to the group and follows the quality principle. Third, groups should not move in a too narrow environment and follow the principle of diversity. Fourthly, groups should avoid changing their behavior with the change of environment and follow the principle of stability. Finally, the behavior of a group can be appropriately changed according to the conditions with low cost.

The development history of swarm intelligence optimization algorithm is shown in Figure 1.

In recent years, the main research aspect is biological swarm intelligence algorithm, and great research results and optimization strategies have also been obtained. The classification diagram of swarm intelligence algorithm is shown in Figure 2.

### 2.2. Particle Swarm Optimization

#### 2.2.1. Basic Concepts

This algorithm is called PSO for short [17, 18], which is developed by researchers through exploring and summarizing the behavior of bird predation. Like birds preying in groups, the optimal solution of this algorithm also needs the cooperation among individual particles. In the process of predation, birds will learn from each other's predation experience, thus forming an exchange of experiences and making the predation process orderly. Similarly, in this algorithm, each particle also needs to realize information exchange, so that the process of finding the optimal solution can be orderly.

*(1) Basic PSO Algorithm*. In a space that needs to be represented by *D* component coordinates, there are countless particles with searching ability. They are not disordered, each particle individual has its own position, and this position is the most suitable position for this individual. PSO algorithm will update the performance of particles according to the velocity update formula. At this time, the intervention of objective function will bring the position comparison before and after the update of particles, which can clearly see whether the updated position is better than the position before the update. Complete the algorithm once in this way. The PSO algorithm flowchart is shown in Figure 3.

The particle iterative update formula is as follows:

(1) $$\begin{array}{c} v_{i}^{t+1}=v_{i}^{t}+c_{1}r_{1}\left(p_{i}^{t}-x_{i}^{t}\right)+c_{2}r_{2}\left(p_{g}^{t}-x_{i}^{t}\right),\\ x_{i}^{t+1}=x_{i}^{t}+v_{i}^{t+1}. \end{array}$$

where *x*_*i*_^*t*^ is the position of the *i*-th particle in the *t*-th iteration, *v*_*i*_^*t*^ is the velocity of the *i*-th particle in the *t*-th iteration, *x*_*i*_^*t*+1^ is the position of the *i*-th particle in the *t*+1 th iteration, *v*_*i*_^*t*+1^ is the velocity of the *i*-th particle in the *t*+1 th iteration, *p*_*i*_^*t*^ indicates the historical optimal position when the *i*-th particle searches to the *t*-th generation, *p*_*g*_^*t*^ is the historical optimal position of the whole population when the *t* generation is searched, that is, the global optimal position, *c*_1_,*c*_2_ is the learning factor, usually 2, and *r*_1_, *r*_2_ is the disturbance factor, usually randomly taken within [0, 1].

The values of C1, C2 and R1, R2 will affect whether the particles rush across the target region or wander outside the target region, and a better solution can be obtained when they are constant values.

The performance of PSO algorithm will influence each other, which leads to the instability of PSO algorithm, so it is necessary to add linear decreasing weights.

The speed update equation at this time is

(2) $$\begin{array}{c} v_{i}^{t+1}=\omega v_{i}^{t}+c_{1}r_{1}\left(p_{i}^{t}-x_{i}^{t}\right)+c_{2}r_{2}\left(p_{g}^{t}-x_{i}^{t}\right). \end{array}$$

The formula of linear decreasing weight strategy is as follows:

(3) $$\begin{array}{c} \omega \left(t\right)=\omega_{\max}-\frac{\omega_{\max}-\omega_{\min}}{G_{\max}}\cdot t, \end{array}$$

where *t* is the current number of iterations, *G*_max_ is the maximum number of iterations, *ω*_max_ is the initial inertia weight, and *ω*_min_ is the inertia weight at the maximum number of iterations *G*_max_, usually 0.4.

*(2) Comprehensive Learning Particle Swarm Optimization Algorithm*. In order to improve PSO algorithm and solve the shortcomings of PSO algorithm, a comprehensive learning strategy is added, and the combination of the two algorithms is developed into CLPSO algorithm. The update speed of CLPSO algorithm is different from that of PSO algorithm [19], and the best position of individuals is an important basis for updating the speed of CLPSO algorithm.

The comprehensive learning particle swarm optimization algorithm firstly calculates the learning probability of each particle *p*_*c*_. The formula is as follows:

(4) $$\begin{array}{c} p_{c_{i}}=a+b*\frac{\exp\left(10*\left(i-1\right)/N-1\right)}{\exp\left(10\right)-1}. \end{array}$$

According to the experimental experience, generally *a* and *b* are constants, usually *a* = 0.05 and *b* = 0.45.

The update formula of comprehensive learning particle swarm optimization algorithm is as follows:

(5) $$\begin{array}{c} v_{id}=w*v_{id}+c*r_{id}\left({\text{pbest}}_{f_{i}\left(d\right),d}-x_{id}\right),\\ x_{id}=x_{id}+v_{id}. \end{array}$$

*Pbest* is the optimal position of the individual. *f*_*i*_(*d*) is the dimension value of the *d* dimension in the best position of the *i*-th particle individual. *f*_*i*_=[*f*_*i*_(1), *f*_*i*_(2),…, *f*_*i*_(*D*)] is the learning sample vector set by particle *i*. *pbest*_*f*_*i*_(*d*),*d*_ indicates the dimension value corresponding to the best position produced by previous iterations of a particle.

Each dimension of the particle will produce a random number and compare the random number with the learning probability parameter *p*_*c*_. If the former is greater than the latter, the dimension of the particle in the best position in each iteration will be learned; otherwise, the dimension of the particle in the best position of the individual will be learned.

Specific subgroup types are as follows:

Extreme learning subgroup:
  (6) $$\begin{array}{c} x_{i}^{t+1}=\left\{\begin{array}{c} \alpha x_{i}^{t}+\beta c_{1}r_{1}\left(g^{t}-x_{i}^{t}\right),\;r\geq p_{g},\\ \alpha x_{i}^{t}+\beta c_{2}r_{2}\left(n^{t}-x_{i}^{t}\right),\;r<p_{g}. \end{array}\right) \end{array}$$
Compound learning subgroup:
  (7) $$\begin{array}{c} x_{i}^{t+1}=\alpha x_{i}^{t}+\beta \left(c_{1}r_{1}\left(g^{t}-x_{i}^{t}\right)+c_{3}r_{3}\left(p_{i}^{t}-x_{i}^{t}\right)\right). \end{array}$$
Domain learning subgroup:
  (8) $$\begin{array}{c} x_{i}^{t+1}=\alpha x_{i}^{t}+\beta c_{2}r_{2}\left(n_{i}^{t}-x_{i}^{t}\right). \end{array}$$
Random learning subgroups:
  (9) $$\begin{array}{c} x_{i}^{t+1}=\alpha x_{i}^{t}+\frac{\beta r_{4}\left(X_{\max}-X_{\min}\right)}{2}. \end{array}$$

The advantage of particle swarm optimization is to avoid the phenomenon that the evolved particles will lose their search ability after many iterations, which makes the algorithm have stronger global search ability and save the calculation times of the algorithm. At the same time, the convergence speed of the comprehensive learning particle algorithm will not lead to the decrease of population diversity, so that the algorithm will not fall into premature convergence, especially for peak and multipeak objective functions. Through the construction of learning application program, the group learning behavior is richer and the diversity of population information is increased.

## 3. Optimization Algorithm

### 3.1. Design of Hybrid Clonal Selection Particle Swarm Optimization

#### 3.1.1. Clone Selection Strategy

In order to improve the PSO, improve the convergence performance, increase the diversity of population, and avoid premature algorithm [20, 21], clonal selection strategy can be combined with PSO [22].

The new population Sub is formed by the expansion and growth of the temporary clone group formed by individual extremum, and the ranking of individuals in the new population will be related to the size of affinity, and the clone size of individual extremum will increase with the increase of affinity. The formula of cloning multiple *N*_*c*_ is as follows:

(10) $$\begin{array}{c} N_{c}=\overset{N}{\underset{i=1}{\sum }}\left(\text{round}\left(\frac{\beta *N}{i+1}\right)*cm\right). \end{array}$$

*N* is Sub scale, *I* is the individual affinity value ranking in Sub, *β* indicates that the cloning coefficient is 0.8, *cm* indicates that the clone cardinality value is 5, and Round represents a function to round an integer.

In Sub population, Cauchy mutation is used to get new mutation individuals, which increases population diversity and improves the global search ability of the algorithm. The mutation operator formula is as follows:

(11) $$\begin{array}{c} x_{ij}\left(t+1\right)=x_{ij}\left(t\right)+r*\text{cauchy}*x_{ij}\left(t\right), \end{array}$$

where *r* is the parameter with a value of 10.

Cauchy variogram is as follows:

(12) $$\begin{array}{c} \text{Cauchy}\left(x\right)=\frac{1}{\pi }*\;\arctan\frac{-0.5+\text{random}\left(\right)*10.0}{t+1}. \end{array}$$

*Random* represents computer-generated random numbers from 0 to 1 and *t* is the number of iterations.

The extreme value of the individual with the highest affinity in the mutated population is compared with the extreme value of the individual in the original population. If the former is higher than the latter, it will be updated and replaced; otherwise, it will remain unchanged. At the same time, the optimal value of individual extremum of population is compared with gbest, and if the former is higher than the latter, it is updated and replaced.

#### 3.1.2. HCSPSO Algorithm Flow

The flowchart of the HCSSPSO algorithm is shown in Figure 4.

#### 3.1.3. Time Complexity Analysis

The time complexity of particle swarm optimization and clonal selection strategy synthesizes the time complexity of HCSSPSO algorithm. The parameter is set as *C* to represent the number of parameters, *T* (*C*) to represent the time complexity of test function, and *O* (*C*).

(13) $$\begin{array}{c} T_{\text{PSO}}\left(C\right)=O\left(\text{Maxlter}*PS*P_{\text{PSO}}*T\left(C\right)\right),\\ T_{\text{CS}}\left(C\right)=O\left(\text{Maxlter}*PS*N_{C}*T\left(C\right)\right),\\ T_{\text{HCSPSO}}\left(C\right)=T_{\text{PSO}}\left(C\right)+T_{\text{CS}}\left(C\right). \end{array}$$

*Maxlter* is the maximum number of iterations of the algorithm, *PS* is the population size, *P*_PSO_ is the individual mutation probability in the algorithm, the value range (0, 1), and *N*_*C*_ is the multiple of particles.

## 4. Simulation Experiment

### 4.1. Convergence Curve

#### 4.1.1. Test Function and Parameter Settings

According to the selected eight test functions, in which functions 1 to 5 are single modal functions and functions 6 to 8 are multimodal functions, the HCSSPSO algorithm, basic PSO algorithm, and CLPSO algorithm are compared, and their ability and convergence speed are analyzed to verify the effectiveness of HCSSPSO algorithm.

Setting parameters: *Gm* = 1000, *pm* = 0.8, *Popsize* = 40, *cm* = 5, *N*_*C*_ = 30.

The 8 standard test functions are as follows:

(14) $$\begin{array}{c} f_{1}\left(x\right)=\overset{D}{\underset{i=1}{\sum }}x_{i}^{2},\;-100\leq x_{i}\leq 100,\\ f_{2}\left(x\right)=\overset{D}{\underset{i=1}{\sum }}{\left(\left|x_{i}+0.5\right|\right)}^{2},\;-100\leq x_{i}\leq 100,\\ f_{3}\left(x\right)=\overset{D}{\underset{i=1}{\sum }}{\left(\overset{2}{\underset{j=1}{\sum }}x_{j}\right)}^{2},\;-100\leq x_{i}\leq 100,\\ f_{4}\left(x\right)=\overset{D}{\underset{i=1}{\sum }}ix_{i}^{4}+\text{random}\left(0,1\right),\;-1.28\leq x_{i}\leq 1.28,\\ f_{5}\left(x\right)=\overset{D}{\underset{i=1}{\sum }}\left|x_{i}\right|+\prod_{i=1}^{D}\left|x_{i}\right|,\;-10\leq x_{i}\leq 10,\\ f_{6}\left(x\right)=\overset{D}{\underset{i=1}{\sum }}\left(x_{i}^{2}-10\;\cos\left(2\pi x_{i}\right)+10\right),\;-5.12\leq x_{i}\leq 5.12,\\ f_{7}\left(x\right)=\frac{1}{400}\overset{D}{\underset{i=1}{\sum }}x_{i}^{2}-\prod_{i=1}^{D}\cos\left(\frac{x_{i}}{\sqrt{i}}\right)+1,\;-300\leq x_{i}\leq 300,\\ f_{8}\left(x\right)=-20\;\exp\left(-0.2\sqrt{\frac{1}{D}\overset{D}{\underset{i=1}{\sum }}x_{i}}\right)-\left(\frac{1}{D}\overset{D}{\underset{i=1}{\sum }}\cos\left(2\pi x_{i}\right)\right)+20+e,\;-32\leq x_{i}\leq 32. \end{array}$$

In this equation, the optimal solution of all functions is set to 0. In comparison, we only compare the overall performance of each algorithm, such as convergence speed, but the overall test of this algorithm is not compared with other algorithms. However, when the whole algorithm has been compared with absolute advantages, and this advantage is in line with the performance of simulation experiments, we think the comparison between the whole test and local advantages can be omitted.

#### 4.1.2. Experimental Comparison and Results

The performance of the algorithm is represented by the mean value and standard deviation of the eight test functions. The convergence rate is reflected by the mean value, while the standard deviation can show the stability of the algorithm. The experimental results are shown in Table 1.

The function includes unimodal function and multimodal function and has a large number of local minima, which can explain the ability of each algorithm to deal with multimodal problems.

It can be seen from the table that the average value and standard value data of HCSSPSO algorithm under 8 evaluation functions are better than the other two algorithms. It can be seen that clonal selection strategy can improve the performance of PSO algorithm and is higher than other optimization algorithms.

The convergence curves of the three algorithms for function 1 are shown in Figure 5.

The convergence curves of the three algorithms for function 2 are shown in Figure 6.

The convergence curves of the three algorithms for function 3 are shown in Figure 7.

The convergence curves of the three algorithms for function 4 are shown in Figure 8.

The convergence curves of the three algorithms for function 5 are shown in Figure 9.

The convergence curves of the three algorithms for function 6 are shown in Figure 10.

The convergence curves of the three algorithms for function 7 are shown in Figure 11.

The convergence curves of the three algorithms for function 8 are shown in Figure 12.

From the above table, we can see that, by comparing the convergence curves obtained from eight classical evaluation functions selected by PSO algorithm, CLPSO algorithm, and HCSSPSO algorithm, we can see that the convergence speed and stability of HCSSPSO algorithm are optimized compared with the other two algorithms and have better optimization ability.

### 4.2. Simulation Experiment and Parameter Setting

#### 4.2.1. Establishment of Objective Function

Community smart sports service for the elderly follows the principle of maximizing benefits, and the elderly judge their satisfaction with smart sports service. Therefore, the use of swarm intelligence algorithm should minimize the allocation cost of community intelligent sports services for the elderly, optimize the service facilities, maximize the satisfaction of the elderly, and maximize the population served. In this experiment, the region is set to N rows and *M* columns, and K smart sports service types are set at the same time. *i* and *j* represent cells (*i*, *j*), N represents total space, Suit represents suitability, and *ω* represents satisfaction. The objective function is as follows:

Service configuration fee:
  (15) $$\begin{array}{c} \text{Min}\overset{n}{\underset{i=1}{\sum }}\overset{m}{\underset{j=1}{\sum }}\overset{k}{\underset{k=1}{\sum }}C_{ijk}N_{ijk}. \end{array}$$
Suitability of service facilities:
  (16) $$\begin{array}{c} \text{Max}\overset{n}{\underset{i=1}{\sum }}\overset{m}{\underset{j=1}{\sum }}\overset{k}{\underset{k=1}{\sum }}{\text{Suit}}_{ijk}N_{ijk}. \end{array}$$
Satisfaction of the elderly:
  (17) $$\begin{array}{c} \text{Max}\overset{n}{\underset{i=1}{\sum }}\overset{m}{\underset{j=1}{\sum }}\overset{k}{\underset{k=1}{\sum }}\omega_{ijk}N_{ijk}. \end{array}$$
Number of serviced population:
  (18) $$\begin{array}{c} \text{Max}\overset{n}{\underset{i=1}{\sum }}\overset{m}{\underset{j=1}{\sum }}\overset{k}{\underset{k=1}{\sum }}\frac{C_{\text{dense}}}{\sum_{i=1}^{n}\sum_{j=1}^{m}\max\left\{\text{dense}\left(c\right)\times D_{\text{area}}\times \;\exp\left(\left[-r\times {\text{dis}}_{x}\left(c\right)\right]\right)\right\}}N_{ijk}. \end{array}$$

*N*_*ijk*_ determine whether the service facility type on cell (*i*, *j*) is equal to *k*, the equal value is 1, and the opposite is 0. dis_*x*_(*c*) represents the Euclidean distance from *C* to *P* communities. dense(*c*) is the Population density on *c*. *D*_area_ is the size of area occupied by service facility type. exp[−*r* × dis_*x*_(*c*)] is the population attraction of *P* community locations to *C*. *C*_dense_ is the objective function coefficient.

#### 4.2.2. Simulation Experiment and Result Analysis

In order to analyze the reasonable feasibility and optimization performance of HCSSPSO algorithm, an optimization model of community intelligent sports service was designed. Firstly, according to the data published by the network, the population density of the elderly in the community is calculated, and all relevant data are converted into parameter data. Assuming that the community service area is 50 × 60 units, according to the survey, the initialization data of community sports service are as follows: service A: 324, service B: 361, service C: 655, service D: 904, service E: 518, and service F: 238. After the algorithm is optimized, the data are as follows: service A: 250, service B: 473, service C: 705, service D: 964, service E: 386, and service F: 222. Publish data through the network, and the evaluation index is the objective function set in 4.2.1. After the data is unified, PSO algorithm, CLPSO algorithm, and HCSSPSO algorithm are applied, and the results are compared. The forecast results are shown in Table 2.

The following is a comparison between the predicted configuration cost, service suitability, satisfaction of the elderly, and service population and the actual values after optimization by PSO algorithm, CLPSO algorithm, and HCSSPSO algorithm, taking a certain 20 days as sampling points in 2020. The data comparison is shown in Table 3.

The actual value of facility cost is compared with the predicted values of three algorithms, such as Figure 13.

The actual suitability values are paired with the predicted values of the three algorithms, such as Figure 14.

The actual value of satisfaction of the elderly is compared with the predicted values of the three algorithms, such as Figure 15.

The actual value of the service population is paired with the predicted values of the three algorithms, such as Figure 16.

Therefore, HCSSPSO algorithm has a higher reasonable degree of resource allocation for community intelligent sports services for the elderly and has higher cost performance, suitability, satisfaction, and even population. Compared with the original data, HCSPOS algorithm greatly optimizes the configuration of community service and brings higher and more advanced community service. Compared with other algorithms, HCSSPSO algorithm is more excellent. Compared with the optimized data, the data obtained by HCSSPSO algorithm is obviously higher than other algorithms. The HCSSPSO algorithm proposed in this paper has more advantages.

## 5. Conclusion

Because PSO algorithm has some shortcomings, it may bring premature problem and cannot guarantee population diversity, so it is not suitable as an algorithm for optimizing intelligent sports. Therefore, this paper proposes HCSSPSO algorithm, which combines PSO algorithm with clonal selection strategy. Compared with PSO algorithm and CLPSO algorithm, it has better convergence speed and stability and is more suitable for resource allocation and optimization of community intelligent sports services for the elderly.

## Figures and Tables

**Figure 1:** Development history of swarm intelligence optimization algorithm.

**Figure 2:** Classification diagram of swarm intelligence algorithm.

**Figure 3:** Flowchart of PSO algorithm.

**Figure 4:** Flowchart of HCSSPO algorithm.

**Figure 5:** Comparison of convergence curves of three algorithms to function 1.

**Figure 6:** Comparison of convergence curves of three algorithms to function 2.

**Figure 7:** Comparison of convergence curves of three algorithms to function 3.

**Figure 8:** Comparison of convergence curves of three algorithms to function 4.

**Figure 9:** Comparison of convergence curves of three algorithms to function 5.

**Figure 10:** Comparison of convergence curves of three algorithms to function 6.

**Figure 11:** Comparison of convergence curves of three algorithms to function 7.

**Figure 12:** Comparison of convergence curves of three algorithms to function 8.

**Figure 13:** Comparison of actual forecast of facility cost.

**Figure 14:** Comparison of actual prediction of suitability value.

**Figure 15:** Comparison of actual predictions of satisfaction of the elderly.

**Figure 16:** Comparison of actual forecast of service population.

**Table 1:** Results of different algorithms in different functions.

Function	Computing mode	PSO	CLPSO	HCSPSO
*f*_1_	Average	0.00017	1.58*E* − 12	1.72*E* − 42
	Standard deviation	0.00026	7.70*E* − 13	2.76*E* − 42
*f*_2_	Average	1.68395	0	0
	Standard deviation	3.88674	0	0
*f*_3_	Average	4101.68	2.56*E* − 01	2.76*E* − 34
	Standard deviation	3820.52	6.38*E* − 01	6.72*E* − 34
*f*_4_	Average	0.04391	5.85*E* − 03	1.20*E* − 06
	Standard deviation	0.01963	1.11*E* − 03	3.67*E* − 06
*f*_5_	Average	7.47418	2.51*E* − 08	1.06*E* − 22
	Standard deviation	6.23788	5.84*E* − 09	1.78*E* − 22
*f*_6_	Average	80.4738	9.09*E* − 05	0
	Standard deviation	22.7835	1.25*E* − 04	0
*f*_7_	Average	0.03571	9.02*E* − 09	4.34*E* − 20
	Standard deviation	0.05439	8.57*E* − 09	2.94*E* − 20
*f*_8_	Average	2.42014	3.66*E* − 07	1.57*E* − 14
	Standard deviation	1.26084	7.57*E* − 08	7.98*E* − 15

**Table 2:** Forecast results.

Objective function	Numerical value			
	Original data	PSO	CLPSO	HCSPSO
Service configuration fee (10,000)	8759.6049	8622.7690	8166.3076	7752.1985
Suitability of service facilities	369855	378860	382491	390167
Satisfaction of the elderly	0.68	0.76	0.81	0.89
Number of service population	23160	24927	25509	26751

**Table 3:** Comparison of actual values and predicted values of the three algorithms.

Sampling time	Category	Actual value	PSO prediction	CLPSO prediction	HCSPSO prediction
1	Facility cost (10,000)	8700	8804	8773	8685
	Suitability	0.56	0.55	0.57	0.59
	Satisfaction of the elderly	0.63	0.55	0.60	0.69
	Number of service population	23106	21045	22621	23891
2	Facility cost (10,000)	8667	8723	8650	8600
	Suitability	0.51	0.43	0.50	0.6
	Satisfaction of the elderly	0.65	0.57	0.60	0.73
	Number of service population	21085	20037	21109	22084
3	Facility cost (10,000)	8623	8876	8732	8540
	Suitability	0.67	0.58	0.65	0.70
	Satisfaction of the elderly	0.70	0.54	0.60	0.73
	Number of service population	27243	25061	24101	29201
4	Facility cost (10,000)	8677	8832	8723	8420
	Suitability	0.70	0.61	0.75	0.79
	Satisfaction of the elderly	0.68	0.60	0.70	0.80
	Number of service population	28347	27140	28897	30142
5	Facility cost (10,000)	8867	9102	8453	8014
	Suitability	0.78	0.69	0.70	0.80
	Satisfaction of the elderly	0.79	0.65	0.70	0.85
	Number of service population	29587	27201	28754	32048
6	Facility cost (10,000)	8593	8804	8675	8103
	Suitability	0.75	0.65	0.71	0.84
	Satisfaction of the elderly	0.82	0.66	0.76	0.88
	Number of service population	28499	26542	27413	30472
7	Facility cost (10,000)	8604	8706	8500	8304
	Suitability	0.84	0.71	0.80	0.91
	Satisfaction of the elderly	0.88	0.72	0.80	0.93
	Number of service population	30139	28046	31284	35041
8	Facility cost (10,000)	8379	8571	8473	8047
	Suitability	0.82	0.70	0.72	0.85
	Satisfaction of the elderly	0.81	0.68	0.76	0.87
	Number of service population	29952	27036	28769	34057
9	Facility cost (10,000)	8508	8934	8764	8204
	Suitability	0.85	0.75	0.80	0.90
	Satisfaction of the elderly	0.87	0.67	0.77	0.93
	Number of service population	32079	30042	31098	35478
10	Facility cost (10,000)	8672	8957	8534	7950
	Suitability	0.80	0.65	0.78	0.85
	Satisfaction of the elderly	0.83	0.71	0.76	0.90
	Number of service population	31085	28014	30795	34258
11	Facility cost (10,000)	8684	8803	8503	8350
	Suitability	0.86	0.76	0.83	0.90
	Satisfaction of the elderly	0.85	0.74	0.81	0.95
	Number of service population	30185	27521	31694	35041
12	Facility cost (10,000)	8578	8954	8764	8046
	Suitability	0.79	0.63	0.75	0.85
	Satisfaction of the elderly	0.80	0.66	0.78	0.89
	Number of service population	30872	27924	29540	36250
13	Facility cost (10,000)	8610	9014	8804	8103
	Suitability	0.88	0.68	0.77	0.94
	Satisfaction of the elderly	0.82	0.72	0.80	0.93
	Number of service population	33105	31024	32680	36572
14	Facility cost (10,000)	8640	8814	8415	7924
	Suitability	0.90	0.80	0.87	0.95
	Satisfaction of the elderly	0.89	0.76	0.84	0.91
	Number of service population	34208	30450	33075	37250
15	Facility cost (10,000)	8796	8924	8821	8430
	Suitability	0.91	0.75	0.80	0.95
	Satisfaction of the elderly	0.89	0.77	0.82	0.91
	Number of service population	35024	34214	36204	38524
16	Facility cost (10,000)	8721	9042	8940	8106
	Suitability	0.90	0.74	0.85	0.96
	Satisfaction of the elderly	0.90	0.77	0.83	0.94
	Number of service population	34802	31064	35014	37562
17	Facility cost (10,000)	8496	8627	8207	7824
	Suitability	0.87	0.68	0.74	0.90
	Satisfaction of the elderly	0.86	0.73	0.90	0.93
	Number of service population	34506	33201	35407	38524
18	Facility cost (10,000)	8143	8524	8410	7731
	Suitability	0.92	0.78	0.90	0.96
	Satisfaction of the elderly	0.93	0.76	0.89	0.97
	Number of service population	35621	30249	35103	38245
19	Facility cost (10,000)	7903	8321	8104	7624
	Suitability	0.91	0.84	0.87	0.93
	Satisfaction of the elderly	0.90	0.74	0.88	0.91
	Number of service population	35102	31259	34520	40641
20	Facility cost (10,000)	7710	8125	7658	7103
	Suitability	0.90	0.82	0.85	0.95
	Satisfaction of the elderly	0.95	0.84	0.90	0.97
	Number of service population	36045	34253	37250	39240

## Data Availability

The experimental data used to support the findings of this study are available from the corresponding author upon request.
